The article "The SDF-1/CXCR4 axis promotes recovery after spinal cord injury by mediating bone marrow-derived from mesenchymal stem cells" was published in 2017. Journal: Oncotarget.

# The SDF-1/CXCR4 axis promotes recovery after spinal cord injury by mediating bone marrow-derived from mesenchymal stem cells

**DOI:** 10.18632/oncotarget.14619

**Published:** 2017-01-13

**Authors:** Guo-Dong Wang, Yi-Xun Liu, Xiao Wang, Yong-Le Zhang, Ya-Dong Zhang, Feng Xue

**Affiliations:** ^1^ Department of Orthopedic, Huaihe Hospital of Henan University, Kaifeng 475000, P.R. China; ^2^ Department of Orthopedic, Shanghai Fengxian Central Hospital, Branch of the Sixth People's Hospital Affiliated to Shanghai Jiao Tong University, Shanghai 201400, P.R. China

**Keywords:** bone marrow-derived mesenchymal stem cells, stromal cell-derived factor-l, chemotaxis cytokine receptor-4, spinal cord injury, hind limb motor function

## Abstract

This study aims to explore the role of the SDF-1/CXCR4 axis in mediating BMSCs and SCI recovery. BMSCs were collected and SCI rat models were established. Wistar rats were assigned into the blank control, sham, SCI, SCI + BMSCs, SCI + BMSCs + SDF-1, SCI + BMSCs + AMD3100 (an inhibitor of SDF-1/CXCR4 axis) and SCI + BMSCs + SDF-1 + AMD3100 groups. Hind limb motor function was measured 7, 14, 21 and 28 days after operation. qRT-PCR, western blotting and ELISA was performed to determine the expressions of SDF-1, CXCR4, NGF, BDNF, GFAP and GAP-43, TNF-α, IL-1β, L-6 and IFN-γ. Hind limb motor function scores 7 days after the operation were reduced in the SCI rats of the blank control and sham groups. Hind limb function was found to be better in the SCI + BMSCs and SCI + BMSCs + SDF-1 groups than in the SCI, SCI + BMSCs + AMD3100 and SCI + BMSCs + SDF-1 + AMD3100 groups 14, 21 and 28 days after operation. Furthermore, the SCI group had lower SDF-1, CXCR4, NGF, BDNF and GAP-43 expressions but higher GFAP, TNF-α, IL-1β, IL-6 and IFN-γ than the blank control and sham groups 28 days after operation. While, the SCI + BMSCs, SCI + BMSCs + SDF-1 and SCI + BMSCs + SDF-1 + AMD3100 groups displayed opposite trends to the SCI and SCI + BMSCs + AMD3100 groups. In conclusion, SDF-1/CXCR4 axis promotes recovery after SCI by mediating BMSCs.

## INTRODUCTION

Spinal cord injury (SCI) is a highly disabling disease which causes disorder loss of sensory and motion function and results in the functional disorders of many other systems such as the respiratory, circulatory, urinary and digestive systems [1, 2]. It is estimated that the morbidity of SCI over the world is about 236 to 1,009 per million [3]. Young adults and male patients are more prone to SCI [1]. The pathology of SCI is mainly broken into primary and secondary SCI. Secondary SCI pathology aggravates the disease and edema, causes degeneration and the necrosis of damaged neurons [4, 5]. At present, SCI treatment is a research hotspot due to its high disability rate and heavy social burden.

The article "The SDF-1/CXCR4 axis promotes recovery after spinal cord injury by mediating bone marrow-derived from mesenchymal stem cells" was published in 2017. Journal: Oncotarget.

Stromal cell-derived factor-l (SDF-l), also called CXCL12, is a chemokine in the CXC family which mediates the chemotactic migration of stem cells, lymphocytes, monocytes and dendritic cells through its interaction with chemotaxis cytokine receptor-4 (CXCR4) [6]. Studies indicate that SDF-l plays an important role in the chemotaxis of stem cells, progenitor cells and organ-specific homing through its interaction with CXCR4 [7–9]. Hypoxic or acidic preconditioning shows that the SDF-1/CXCR4 axis has a therapeutic potential in animal models and progenitor cell functions *in vitro* [7]. Interestingly, the SDF-1/CXCR4 axis is critical for the apoptosis, migration and cytokine secretion of bone marrow mesenchymal stem cells (BMSCs) [8]. Adult BMSCs in bone marrow have multiple functions and can migrate to damaged tissue and chronic inflammatory sites [10]. A number of pre-clinical animal studies show that BMSCs transplanted *in vivo* can migrate to damage bone and cartilage sites. In addition, BMSCs transplants can promote the repair of lung damage, liver damage, local limb ischemia and skin injury [11–15]. A variety of proteins such as bone morphogenic protein, epidermal growth factor, transforming growth factor, SDF, tumor necrosis factor and hemolytic pity fatty acid receptor were detected on the surface of the BMSCs [16]. This indicates that the interaction of SDF-1 and CXCR4 has a significant regulatory role in the migration of BMSCs and acute pancreatitis [17]. Another study reported that erythropoietin mobilizes BMSCs to the lesion site post SCI. This promotes the anti-apoptotic effects of BMSCs by enhancing the expression of the SDF-1/CXCR4 axis [18]. Therefore, we hypothesize that the SDF-1/CXCR4 axis is involved in SCI by mediating BMSCs.

## RESULTS

### Observation and identification of BMSCs through an electron microscope and flow cytometry assay

The primary BMSCs were round or oval in shape and the cell pseudopodia displayed clone-like growth after being cultured for 3 days. On the 7th day of cell cultivation, the cells covered the sides of the bottle and were closely interlaced. The results of flow cytometry assay showed a positive stem cell surface rate as the markers CD29 and CD90 were more than 99%. The hematopoietic stem surface markers CD34 and CD45 were less than 2%. This demonstrates that the cell samples are suitable for further experiments (Figure 1).

**Figure 1:** Observation of BMSCs through an electron microscope and flow cytometry assay Note: **(A)** electron microscope photograph of cell 3 and 7 days after cultivation; **(B)** flow cytometry diagram of surface antigens; BMSCs, bone marrow-derived mesenchymal stem cells.

The article "The SDF-1/CXCR4 axis promotes recovery after spinal cord injury by mediating bone marrow-derived from mesenchymal stem cells" was published in 2017. Journal: Oncotarget.

### Living condition and weight changes of rats in each group

After the rats recovered from anesthesia, the rats in the blank control group presented normal physiological functions, while the rats in the sham group were abnormal in walking, this phenomenon was completely recovered 1 d after operation. The rats in the SCI, SCI + BMSCs, SCI + BMSCs + SDF-1, SCI + BMSCs + AMD3100 and SCI + BMSCs + SDF-1 + AMD3100 groups had symptoms including edema of spinal cord, ischemia, paralysis of hind limb, involuntary spastic swing of small amplitude in rat tail; and spasm, curl, high tension and twitch were also found after rat tail was pressed by fingers. In the process of model establishment, 4 rats died from infection and bladder rupture (8% mortality rate), thus only 9 rats were available in each group for further experimentation. There was no significant difference in rat weight between the blank control and sham groups, and the rat's weight increased steadily with time (*P* > 0.05). In comparison to the sham group, the weight of the rats in the SCI, SCI + BMSCs, SCI + BMSCs + SDF-1, SCI + BMSCs + AMD3100 and SCI + BMSCs + SDF-1 + AMD3100 groups had no significant difference 7 days after model establishment. However, weight decreased significantly on the 14th, 21st and 28th day (*P* < 0.05). In comparison to the SCI group, no significant difference was observed in the SCI + BMSCs + AM3100 group. The rats’ weight in the SCI + BMSCs, SCI + BMSCs + SDF-1 and SCI + BMSCs + SDF-1 + AMD3100 groups increased significantly, among which the SCI+BMSCs+SDF-1 group's weight increased more compared to the SCI + BMSCs and SCI + BMSCs + SDF-1 + AMD3100 groups (*P* < 0.05). No significant difference was observed when comparing to the sham group (*P* > 0.05). The SCI + BMSCs group had no significant difference compared with the SCI + BMSCs + SDF-1 + AM3100 group at any time interval (*P* > 0.05) (Table 1).

**Table 1:** Weight (g) changes in the rat models among the blank control, sham, SCI, SCI + BMSCs, SCI + BMSCs + SDF-1, SCI + BMSCs + AMD3100 and SCI + BMSCs + SDF-1 + AMD3100 groups

Groups	7th d	14th d	21th d	28th d
Blank control	221 ± 7	225 ± 4	229 ± 6	233 ± 7
Sham	221 ± 7	225 ± 4	229 ± 6	233 ± 7
SCI	218 ± 7	210 ± 5^a^	200 ± 7^a^	194 ± 7^a^
SCI + BMSCs	219 ± 7	213 ± 7^a b^	204 ± 7^ab^	199 ± 7^ab^
SCI + BMSCs + SDF-1	220 ± 7	218 ± 7^abc^	213 ± 7^bc^	209 ± 7^bc^
SCI + BMSCs + AM3100	219 ± 7	214 ± 7^a^	205 ± 7^a^	200 ± 7^a^
SCI + BMSCs + SDF-1 + AMD3100	219 ± 7	216 ± 7^ab^	207 ± 7^ab^	202 ± 7 ^ab^

BMSCs, bone marrow-derived mesenchymal stem cells; SCI, spinal cord injury; SDF-1, Stromal cell-derived factor-l; ^a^compared with the blank control and Sham groups, *P* < 0.05; ^b^compared with the SCI and SCI + BMSCs + AM 3100 groups, *P* < 0.05; ^c^compared with the SCI + BMSCs and SCI + BMSCs +SDF-1+ AM 3100 groups, *P* < 0.05.

The article "The SDF-1/CXCR4 axis promotes recovery after spinal cord injury by mediating bone marrow-derived from mesenchymal stem cells" was published in 2017. Journal: Oncotarget.

### Comparison of rat hind limb motor function in each group

Scores of the modified Tarlov scale, BBB scale and modified inclined plate test are displayed in Figure 2. In comparison to the blank control and sham groups, the BBB scale scores of the five groups were decreased on the 7th day after model establishment (*P* < 0.05). The relevant operation was performed on the 7th day and the scores of the modified Tarlov scale, BBB scale and modified inclined plate test of the BMSCs and BMSCs + SDF-1 groups were significantly higher than the SCI, SCI + BMSCs + AMD3100 and SCI + BMSCs + SDF-1 + AMD3100 groups on the 14th, 21st and 28th day (*P* < 0.05). The SCI + BMSCs + SDF-1 group had higher scores in the modified Tarlov scale, BBB scale and modified inclined plate than the SCI + BMSCs group (*P* < 0.05). However, there was no difference when comparing to the sham group (*P* *>* 0.05). The SCI + BMSCs group had no significant difference to the SCI + BMSCs + SDF-1 + AM3100 group at any time interval (*P* > 0.05).

**Figure 2:** Comparison of hind limb motor function over time among the blank control, sham, SCI, SCI + BMSCs, SCI + BMSCs + SDF-1, SCI + BMSCs + AMD3100 and SCI + BMSCs + SDF-1 + AMD3100 groups Note: **(A)** a modified Tarlov scare score picture of hind limb motor function; **(B)** modified inclined plate test picture of hind limb motor function; **(C)** BBB locomotor scale score picture of hind limb motor function; BBB, Basso, Beattie and Bresnahan; BMSCs, bone marrow-derived mesenchymal stem cells; SCI, spinal cord injury; SDF-1, Stromal cell-derived factor-l.

### Comparison of inflammatory reaction of rats in each group

The inflammatory reaction in the SCI, SCI + BMSCs, SCI + BMSCs + SDF-1, SCI + BMSCs + AMD3100 and SCI + BMSCs + SDF-1 + AMD3100 groups were enhanced compared to the blank control and sham groups at the early stage of SCI. On the 14th day after model establishment, a large amount of inflammatory cell infiltration, obvious edema and congestion phenomenon was observed in the gray substance of spinal cord in the SCI, SCI + BMSCs, SCI + BMSCs + SDF-1, SCI + BMSCs + AMD3100 and SCI + BMSCs + SDF-1 + AMD3100 groups. On the 21st and 28th day after model establishment, the SCI and BMSCs + SDF-1 + AMD3100 groups displayed partial neuron denaturation, degeneration, and even necrosis cysts. The arrangement of nerve fibers was loose and irregular in the white substance of the spinal cord. Tissue structures of the SCI + BMSCs + SDF-1 + AMD3100 groups were relatively complete and clear. The inflammatory reaction in the SCI + BMSCs and SCI + BMSCs + SDF-1 groups reduced significantly and no there were no obvious necrosis cysts. In the SCI + BMSCs + SDF-1 group, neuranagenesis was very clear (Figure 3).

The article "The SDF-1/CXCR4 axis promotes recovery after spinal cord injury by mediating bone marrow-derived from mesenchymal stem cells" was published in 2017. Journal: Oncotarget.

**Figure 3:** Comparison of the inflammatory reaction 28 days after model establishment detected through HE staining among the blank control, sham, SCI, SCI + BMSCs, SCI + BMSCs + SDF-1, SCI + BMSCs + AMD3100 and SCI + BMSCs + SDF-1 + AMD3100 groups Note: HE, hematoxylin and eosin; BMSCs, bone marrow-derived mesenchymal stem cells; SCI, spinal cord injury; SDF-1, Stromal cell-derived factor-l.

### Comparison of mRNA expressions of rats in each group

The mRNA expression of the SDF-1, CXCR4, NGF, BDNF and GAP-43 groups decreased significantly, whereas GFAP increased significantly in the SCI, SCI + BMSCs, SCI + BMSCs + AMD3100 and SCI + BMSCs + SDF-1 + AMD3100 groups (*P* < 0.05) when compared to the blank control and sham groups. No significant difference was observed in the SCI + BMSCs + SDF-1 groups (*P* > 0.05). The SCI + BMSCs + SDF-1, SCI + BMSCs and SCI + BMSCs + SDF-1 + AMD3100 groups had an increased mRNA expression of SDF-1, CXCR4, NGF, BDNF and GAP-43 but decreased GFAP expression (*P* < 0.05) compared to the SCI group. In comparison to the SCI + BMSCs group, the SCI + BMSCs + SDF-1 + AMD3100 group displayed no significant difference (*P* > 0.05); whereas the SCI + BMSCs + SDF-1 group had an increased mRNA expression of SDF-1, CXCR4, NGF, BDNF and GAP-43 and decreased GFAP expression (*P* < 0.05) (Figure 4).

**Figure 4:** Comparison of the mRNA expression of SDF-1, CXCR4, NGF, BDNF, GFAP and GAP-43 detected using qRT-PCR among the blank control, sham, SCI, SCI + BMSCs, SCI + BMSCs + SDF-1, SCI + BMSCs + AMD3100 and SCI + BMSCs + SDF-1 + AMD3100 groups Note: SDF-1, stromal cell-derived factor-1; CXCR4, chemokine receptor-4; GFAP, glial fibrillary acidic protein; GAP-43, Growth associated protein-43; NGF, Nerve growth factor; BDNF, brain derived neurotrophic factor; BMSCs, bone marrow-derived mesenchymal stem cells; SCI, spinal cord injury; SDF-1, Stromal cell-derived factor-l; qRT-PCR, quantitative real-time polymerase chain reaction; acompared with the blank control and sham groups, P < 0.05; bcompared with the SCI and SCI + BMSCs + AM 3100 groups, P < 0.05; ccompared with the SCI + BMSCs and SCI + BMSCs +SDF-1+ AM 3100 groups, P < 0.05.

### Comparison of protein expressions of rats in each group

The protein expression of SDF-1, CXCR4, NGF, BDNF, GFAP and GAP-43 28 days after model establishment detected through western blotting is shown in Figure 5. In comparison to the blank control and sham groups, the protein expression of SDF-1, CXCR4, NGF, BDNF and GAP-43 decreased significantly while GFAP increased significantly in the SCI, SCI + BMSCs, SCI + BMSCs + AMD3100 and SCI + BMSCs + SDF-1 + AMD3100 groups (*P* < 0.05). No significant difference was observed in the SCI + BMSCs + SDF-1 group (*P* > 0.05). Compared with the SCI group, the SCI + BMSCs + SDF-1, SCI + BMSCs and SCI + BMSCs + SDF-1 + AMD3100 groups had increased protein expressions of SDF-1, CXCR4, NGF, BDNF and GAP-43, but a decreased GFAP expression (*P* < 0.05). No significant difference was observed in the SCI + BMSCs + AMD3100 group (*P* > 0.05). There was no significant difference between the SCI + BMSCs group and the SCI + BMSCs + SDF-1 + AMD3100 group (*P* > 0.05). However, the SCI + BMSCs + SDF-1 group had significantly higher protein expressions of SDF-1, CXCR4, NGF, BDNF and GAP-43 but lower GFAP expression (*P* < 0.05) when compared to the SCI + BMSCs group.

The article "The SDF-1/CXCR4 axis promotes recovery after spinal cord injury by mediating bone marrow-derived from mesenchymal stem cells" was published in 2017. Journal: Oncotarget.

**Figure 5:** Comparison of the protein expression of SDF-1, CXCR4, NGF, BDNF, GFAP and GAP-43 detected through western blotting among the blank control, sham, SCI, SCI + BMSCs, SCI + BMSCs + SDF-1, SCI + BMSCs + AMD3100 and SCI + BMSCs + SDF-1 + AMD3100 groups Note: SDF-1, stromal cell-derived factor-1; CXCR4, chemokine receptor-4; GFAP, glial fibrillary acidic protein; GAP-43, Growth associated protein-43; NGF, Nerve growth factor; BDNF, brain derived neurotrophic factor; BMSCs, bone marrow-derived mesenchymal stem cells; SCI, spinal cord injury; SDF-1, Stromal cell-derived factor-l; acompared with the blank control and sham groups, P < 0.05; bcompared with the SCI and SCI + BMSCs + AM 3100 groups, P < 0.05; ccompared with the SCI + BMSCs and SCI + BMSCs +SDF-1+ AM 3100 groups, P < 0.05.

### Comparison of rat inflammatory cytokines expression in each group

The expression of TNF-α, IL-1β, IL-6, IFN-γ 28 days after model establishment was detected using ELISA. These results are presented in Figure 6. The expression of TNF-α, IL-1β, IL-6, IFN-γ increased significantly more in the SCI, SCI + BMSCs, SCI + BMSCs + AMD3100 and SCI + BMSCs + SDF-1 + AMD3100 groups (*P* < 0.05) than the blank control and sham groups. No significant difference was observed in the SCI + BMSCs + SDF-1 group (*P* > 0.05). Compared with the SCI group, the SCI + BMSCs + SDF-1, SCI + BMSCs and SCI + BMSCs + SDF-1 + AMD3100 groups had decreased expressions of TNF-α, IL-1β, IL-6, IFN-γ (*P* < 0.05). No significant difference was observed in the SCI + BMSCs + AMD3100 group (*P* > 0.05). The SCI + BMSCs + SDF-1 + AMD3100 group had no significant difference compared to the SCI + BMSCs group (*P* > 0.05), however, the SCI + BMSCs + SDF-1 group had a decreased protein expression of TNF-α, IL-1β, IL-6, IFN-γ (*P* < 0.05).

The article "The SDF-1/CXCR4 axis promotes recovery after spinal cord injury by mediating bone marrow-derived from mesenchymal stem cells" was published in 2017. Journal: Oncotarget.

**Figure 6:** Comparison of inflammatory cytokines expression using ELISA among the blank control, sham, SCI, SCI + BMSCs, SCI + BMSCs + SDF-1, SCI + BMSCs + AMD3100 and SCI + BMSCs + SDF-1 + AMD3100 groups Note: TNF-α, tumor necrosis factor-α; IL-1β, interleukine-1β; IL-6, interleukine-6; IFN-γ, interferon-γ; ELISA, enzyme-linked immunosorbent assay; BMSCs, bone marrow-derived mesenchymal stem cells; SCI, spinal cord injury; SDF-1, stromal cell-derived factor-l; acompared with the blank control and sham groups, P < 0.05; bcompared with the SCI and SCI + BMSCs + AM 3100 groups, P < 0.05; ccompared with the SCI + BMSCs and SCI + BMSCs +SDF-1+ AM 3100 groups, P < 0.05.

## DISCUSSION

A comparison of the improved Tarlov, inclined plate and BBB scale results demonstrate that BMSCs can promote the repair of SCI through the interaction of SDF-1 with its receptors. The BBB rating is one of the most frequently used assessment methods to evaluate the motor function of rats with SCI. It utilizes 21 levels to observe hind limb activities including the number and range of the activity of each joint of the hind legs, the ability to support the body and the coordination between the forelimb and hind limbs [19]. The modified Tarlov and inclined plate tests are also often used to assess motor function [20–22]. In a recent study, motor function was assessed at different time points after modeling using the BBB rating, inclined plane test and improved Tarlov score [23].

When compared with the blank control and sham groups, the expressions of SDF-1, CXCR4, NGF, BDNF and GAP-43 decreased while GFAP expression increased in the SCI, SCI + BMSCs, SCI + BMSCs + AMD3100 and SCI + BMSCs + SDF-1 + AMD3100 groups. Furthermore, it was found that the SCI + BMSCs + SDF-1 group had an increased expression of SDF-1, CXCR4, NGF, BDNF and GAP-43 but decreased GFAP expression compared to the SCI + BMSCs group. This indicates that the SDF-1/CXCR4 axis promotes the expression of SDF-1, CXCR4, NGF, BDNF via mediating BMSCs. SDF-1 attracts immune cells and endogenous precursor/stem cells to the injured site and enhances axonal sprouting after SCI [24]. Neurotropic factors such as BDNF and NGF play crucial roles in nerve regeneration after SCI [25]. Pretreatment with electroacupuncture promotes the production of BDNF and SDF-1α which exerts a protective effect on focal cerebral ischemia [26]. The binding of SDF-1 to CXCR4 induces osteoarthritic cartilage degeneration and these catabolic processes can be disrupted by a pharmacologic blockade of SDF-1/CXCR4 signaling [27]. Chen et al. indicated that NGF provides a synergistic effect in the treatment of SCI in rats which promotes functional recovery and neural regeneration [28]. A large number of pre-clinical animal studies have shown that transplanted BMSCs *in vivo* can migrate to the defective area of bone and cartilage, myocardial infarction or cerebral ischemia areas to promote the repair of lung damage, liver damage, limb ischemia and skin damage [12, 13, 15, 29]. Interestingly, allogeneic BMSCs transplantation is effective in stimulating the recovery of spinal cord function in rats with SCI. In addition, the optimal time of BMSCs transplantation is 3 days after injury [30]. Ritfeld et al. found that BDNF dependency can enhance anatomical spinal cord repair [31].

The article "The SDF-1/CXCR4 axis promotes recovery after spinal cord injury by mediating bone marrow-derived from mesenchymal stem cells" was published in 2017. Journal: Oncotarget.

Importantly, the SDF-1/CXCR4 axis promoted GAP-43 expression and lowered GFAP expression during SCI repair. GAP-43 participates in the regulation of actin cytoskeleton dynamics in the neuronal axon terminals [32]. GAP-43-labeled axons are able to penetrate and infiltrate damaged tissue and immunoreactivity is significantly higher in re-growing axons and cell bodies within the central lesion cavity [33]. A previous study demonstrated that ephrinB3 silencing enhances axonal growth regeneration and promotes recovery from SCI by significantly increasing the expression of GAP-43 [34]. Another study suggested that the expression of GAP-43 mRNA and protein may be up-regulated after brachial plexus injury, and that GAP-43 protein is associated with function reconstruction and axon regeneration [35]. GFAP is expressed in the central nervous system [36]. Reducing GFAP expression seems to attenuate astrocyte reactivation which may be beneficial for neuronal survival [37]. Cells transplanted in the periphery of the lesion together with GFAP-positive astrocytes have been reported to lead to a significant reduction of GFAP staining intensity [38]. Jin et al. also found that a decreased GFAP expression around the lesion in both the human glial-restricted progenitors (hGRP) and astrocytes derived from hGRP groups relate to the control injury group. This indicates a dramatic inhibition of scar formation [39]. To move forward, Luo et al. suggested that in spinal cord neural development, SDF1 alpha can modulate the migration of progenitor cells through a CXCR4 signaling pathway [40]. As a whole, we analyzed the expression of GAP-43 and GFAP in other recovery processes. We reached the conclusion that SDF-1 promotes GAP-43 expression and lowers GFAP expression during SCI repair.

Furthermore, the SDF-1/CXCR4 axis reduces inflammatory reaction induced by SCI via BMSCs. Measuring serum levels of TNF-α and IL-1β over time could be important to track the course of SCI [41]. TNF-α expression is significantly promoted in rats with SCI, however, it is suppressed after rituximab treatment. The expression of IL-1β and IL-6 are both increased in glial cells without any significant change after rituximab administration [42]. Flavopiridol nanoparticles significantly decrease inflammatory factor synthesis by astrocytes such as TNF-α, IL-1β, and IL-6. This is to decrease cell-cycle activation, facilitate neuronal survival and regeneration, glial scarring, and inflammatory expression [43]. Geng CK et al. demonstrated that by decreasing TNF-α, IL-1β, IL-6 and IFN-α, BMSCs transplantation can promote the functional recovery of rat hind limbs after SCI [44].

The article "The SDF-1/CXCR4 axis promotes recovery after spinal cord injury by mediating bone marrow-derived from mesenchymal stem cells" was published in 2017. Journal: Oncotarget.

In addition, the SDF-1/CXCR4 axis can enhance recovery after SCI by mediating BMSCs.There is, however, a limitation in the present study. The sample size is limited and the specific interaction mechanism of BMSCs with SDF-1 and CXCR4 is still in need of further exploration.

## MATERIALS AND METHODS

### Ethical statement

The present study was approved by the animal ethics committee and was conducted in accordance to the relevant agreements with the Huaihe Hospital of Henan University.

### Experimental animals

A total of 80 male Wistar rats (200–220 g) at 7 weeks of age were purchased from Beijing FHK bioscience Co. Ltd (Beijing, China). All rats were fed in the SPF laboratory separately at a room temperature of 25 ± 3^°^C and a relative humidity of 55%~75%. The rats had free access to food and water which underwent ultraviolet disinfection and the cages were changed every two days. BMSCs were extracted from 10 rats, 10 rats in the blank control group did not undergo any operation, 10 were used as a sham group and the remaining 50 for model establishment.

### BMSCs culture and preparation

Under aseptic, the thigh bone was separated and washed using Dulbecco's modified eagle medium (DMEM/F12). Fresh bone marrow was extracted and subsequently monocytes were obtained using gradient centrifugation. Separated monocytes were seeded in a 10% fetal bovine serum (Gibco, CA, USA). Penicillin 0.1 U/L and streptomycin 0.1 U/L (Sigma, MO, USA) was added into the DMEM solution and then cultivated at 37^°^C with 5% CO_2_. The solution was changed every two days until reaching approximately an 80–90% confluence level. Surface antigens were detected using flow cytometry assay when the density of BMSCs grew to 60%~70% in confluence. Cell suspension was digested using 0.25% trypsin and the antibodies of CD29, CD90, CD34 and CD45 (Abcam, MA, USA), and then was incubated at room temperature for 30 min. The cells with positive CD29 and CD90 but negative CD34 and CD45 were verified as BMSCs. These cells were diluted (1 × 10^5^ cells/mL) for further experiments.

The article "The SDF-1/CXCR4 axis promotes recovery after spinal cord injury by mediating bone marrow-derived from mesenchymal stem cells" was published in 2017. Journal: Oncotarget.

### Establishment of SCI rat models

For adaptation a total of 50 rats (aged 7 weeks) were fed 2 for weeks. Subsequently, they were anaesthetized using chloral hydrate and the Allen method was utilized. The SD rats were fixed on the operating table in a prone position and the exact location of the T10 segment was marked out. A surgical knife was used to cut a longitudinal skin incision (4 cm) to expose the subcutaneous tissue, deep fascia, muscle, and spinous process of T10. A small bone forcep was used to remove the rat's spinal processes and lamina of the T10 and then they were modified into bony windows with the spinal dural sac exposed. A plastic gasket (3 mm) was then placed on the T10 and a Kirschner wire (10 g; 2.5 mm in diameter of the bottle) was dropped on the T10 to make cause a blast injury. The site of injury was congested accompanied with edema rapidly. After rat models with SCI were established, iodophor and physiological saline was used to wash the spinal cord. Antibiotics were partially dropped and then the muscle, fascia and skin were sewed step by step. After surgery, an intraperitoneal injection of penicillin (200,000 U/time) was injected for 7 days. Lower abdominal pressure was applied to the rat's bladder to force urination 2 times per day until they could naturally urinate. Rat models with limb paralysis were then established.

### Animals grouping

Rats were divided into several groups (nine rats each group): (1) blank control group (healthy rats without any treatment); (2) sham group (healthy rats treated using a sham-operation); (3) SCI group (SCI rats without any treatment); (4) BMSCs group (SCI rats treated using 5 μL BMSCs); (5) BMSCs + SDF-1 group (SCI rats treated using 5 μL BMSCs plus 1μg SDF-1); (6) BMSCs + AMD3100 (an inhibitor of SDF-1/CXCR4 axis) group (SCI rats treated using 5 μL BMSCs plus 1 μg AMD3100); (7) BMSCs + SDF-1 + AMD3100 group (SCI rats treated using 5 μL BMSCs + 1 μg SDF-1 + 1 μg AMD3100). Appropriate treatment began 7 days after surgery and the corresponding processing reagents were intrathecally injected at the lumbar spine every 2 days. The control group was injected with 1 mL saline and the other groups had corresponding reagent injections. Protein SDF-1α 1 μg and CXCR4 antagonists 1 μg (purchased from R&D, MN, USA) were intrathecally injected at the lumbar cord every 2 days. A 1 mL BMSCs mixture was also injected once a day. The experiment lasted 28 days.

### Motor function assessment scales

Hind limb motor function of the rats in each group was assessed using the Basso, Beattie and Bresnahan (BBB) assessment scales 7 days, 14 days, 21 days and 28 days after model establishment. The weight of each rat was also measured. Rats were kept in an open space (125 cm × 125 cm) which allowed free movement. By luring rats with goods, we observed and assessed the relevant indicators of hind limb motor function and physical control function for 4 min. The standard for the modified Tarlov scare score is: 0 points, hind limb had no activity or ability to load; 1 point, hind limb had little activity but no ability to load; 2 points, hind limb had frequent activity but no ability to load; 3 points, hind limb had the ability to load and walk 1–2 steps; 4 points, rat was able to walk with only a slight impairment; 5 points, rat could walk naturally. Under the modified inclined plate standard: rat bodies were fixed with its axis vertical on the inclined plate. The inclined plate test was conducted: plate raised 5 degrees each time and the function value was measured as rats could stay at the maximum angle for 5 s. In the BBB scale, hind limb motor function is divided into 22 levels: 0 for totally paralysis, 21 points for completely normal action, and 1~20 is relevantly identified according to the rating details, which can be found in the records of previous literature in three sections [45]. The first section mainly assesses the flexibility degree and motion details of hind limb joints. The second section assesses the gait and coordination of hind limbs. The third section assesses rat toe fine motor function.

The article "The SDF-1/CXCR4 axis promotes recovery after spinal cord injury by mediating bone marrow-derived from mesenchymal stem cells" was published in 2017. Journal: Oncotarget.

### Hematoxylin and eosin (HE) staining

After BBB assessment, three rats in each group were euthanized and their spinal cord tissue was fixed using 4% paraformaldehyde to create 10 mg specimens. Subsequently, the remaining spinal cord was quick frozen using liquid nitrogen and stored in a refrigerator at –80^°^C. The spinal cords were then cut into slices (10 μm in thickness) along the longitudinal axis of the spinal cord. These were then patched and fixed on a glass slide with polylysine. After being dyed with hematoxylin and eosin, the slices were observed under a fluorescence microscope with a 350 nm wave length. The operations were as follows: the frozen slices were fixed at 4^°^C using precooled acetone for 2 min and then washed with water for 1~2 s. Subsequently, hematoxylin was added, the glass slide was incubated at room temperature for 5 min and then slowly rewashed with water for 5–10 min. The slices were soaked in 1% hydrochloric acid for about 5~10 s and then washed for 2 min using distilled water twice. The slices were then dyed using eosin again for 1–2 min and then rewashed using distilled water for 1~2 s. The slices had a dehydration gradient of 80%, 90% and 100% ethanol. Each gradient lasted for 30 s. Finally, they were soaked in xylene I and II for 5 min and sealed with neutral gum.

The article "The SDF-1/CXCR4 axis promotes recovery after spinal cord injury by mediating bone marrow-derived from mesenchymal stem cells" was published in 2017. Journal: Oncotarget.

### Quantitative real-time polymerase chain reaction (qRT-PCR)

After spinal cord cells were digested and cells lysed, total RNA was isolated from cells according to the kit instructions (CAS: 74104; QIAGEN, Valencia, CA). A total of 5 μL of RNA from each group was obtained and ultra-pure water of RNA enzyme was added to dilute the substance at a ratio of 1:20. The OD260/280 value was measured using ultraviolet spectroscopy and RNA concentration and purity was also calculated. The rate of OD 260/280 was confirmed to be between 1.8~2.0 to ensure the purity of RNA. Agarose gel electrophoresis (1%) was also conducted to uphold integrity. Reverse transcription was performed according to the Fermentas kit instructions. The amplification conditions were denaturation at 95°C for 20 s, annealing at 55°C for 30 s, and extension at 72°C for 40 s, for a total of 40 cycles. Primer 5.0 software was used for primer design. GAPDH was implemented as the internal control, the sequences of primers are presented in Table 2. Ct was obtained and then 2^–ΔΔCt^ was used for quantitative analysis of the mRNA expression of SDF-1, CXCR4, NGF, BDNF, GFAP and GAP-43.

**Table 2:** The primer sequences for quantitative real-time polymerase chain reaction

Gene	Sequence
SDF-1	F: AAA AGA ATT CAT GAA CGC CAA GGT CGT G
	R: AAA GGT ACC ATC TTG AAC TTG TTT AAA G
CXCR4	F: GGG CTG GAG AGC GAG CAT TGC
	R: ATC GGC GAA GAT GTC GGC CT
NGF	F: CGG TCT TCC CGC CCT AGC CTG
	R: ATT TGC ACG CCG CTC CTT TGC
BDNF	F: AGA GTG ATG ACC ATC CTT TT
	R: ATC CAC TAT CTT CCC CTT TT
GFAP	F: GCT AAT GAC TAT CGC CGC CAA CT
	R: CTC CTT AAT GAC CTC GCC ATC CC
GAP-43	F: GGA GGG AGA TGG CTC TGC TAC
	R: AGT GAC AGC AGC AGG CAC ATC
GAPDH	F: AAG GTC ATC CCA GAG CTG AAC GG
	R: ACA ACC TGG TCC TCA GTG TAG CC

SDF-1, stromal cell-derived factor-1; CXCR4, chemokine receptor-4; NGF, nerve growth factor; BDNF, brain derived neurotrophic factor; GFAP, glial fibrillary acidic protein; GAP-43, growth associated protein-43; qRT-PCR, quantitative real-time polymerase chain reaction; F, forward; R, reverse.

### Western blotting

After washing with phosphate buffered saline (PBS) and the appropriate amount of cell lysates was added, the spinal cord tissues were shaken at 4°C for 5 min and centrifuged at 4°C for 10 min (12000 × g). The supernatant was collected and protein was extracted using the Qproteome Mammalian Protein Prer kit (QIAGEN, GmbH, Germany). Once the corresponding protein concentration was detected and trimmed, burning and a total of 6 × buffer was added and stored at –20°C. The 50 μg of protein was conducted using sodium dodecyl sulfate-polyacrylamide gel electrophoresis (SDS-PAGE) electrophoresis and was transferred to a nitrocellulose filter (NC filter) using a siphon action. After sealing with skimmed milk, the mouse anti-human monoclonal antibodies GAP-43, SDF-1, CXCR4, NGF, BDNF and GFAP (1:200) were added to the protein and incubated overnight. TBST was used to wash the membrane 4 times for 10 min each time and the substrate was used. After adding goat anti-mouse IgG (1:10000) tagged with IRDyeTM800DX they were incubated at room temperature for 1 h. All antibodies were purchased from Upstate Biotechnology, Inc. (NY, USA). Protein bands were analyzed and processed using the LabWorks Image Acquisition and Analysis Software (UVP, Inc., Upland, CA, USA) to obtain the relevant protein concentration.

The article "The SDF-1/CXCR4 axis promotes recovery after spinal cord injury by mediating bone marrow-derived from mesenchymal stem cells" was published in 2017. Journal: Oncotarget.

### Enzyme-linked immunosorbent assay (ELISA)

The previously frozen spinal cord tissue which was stored at –80°C was unfrozen using an ultrasonic homogenization ice bath (3 mL lysate/g). After 20 min at 4°C, it was centrifuged for 15 min at 3000 r/min. The liquid supernatant was extracted and other standard samples of varying concentrations (100 μL/well) were detected according to the instructions of the ELISA kit (Hoffmann-La Roche Ltd., Basel, Switzerland). OD (A) value was tested on the wavelength of 450 nm using an Elecsys2010 (Hoffmann-La Roche Ltd., Basel, Switzerland).

### Statistical method

SPSS19.0 statistical software was used to analyze the data. Measurement data was expressed as mean ± standard deviation (SD). The comparison between two group averages was performed using the *t*-test. The comparison of multiple groups was performed using One-Way ANOVA analysis (uniformity test of error variance before analysis). The pairwise comparison of many groups was performed using the LSD-*t* test. Bilateral *P* < 0.05 was considered statistically significant.
